# Effect of Different Ankle-Foot Immobility on Lateral Gait Stability in the Stance Phase

**DOI:** 10.1155/2022/7135040

**Published:** 2022-08-03

**Authors:** Wen Fan, Yasuhiko Hatanaka

**Affiliations:** ^1^Graduate School of Health Science, Suzuka University of Medical Science, 5100293 Mie, Japan; ^2^Department of Rehabilitation Physical Therapy Course, Faculty of Health Science, Suzuka University of Medical Science, 5100293 Mie, Japan

## Abstract

**Background:**

This study aimed to investigate the effect of limited foot and ankle mobility on the lateral stability of gait through the observation of the mediolateral margin of stability and related kinematic parameters.

**Methods:**

Thirty young, healthy participants walked at a fixed gait velocity on a level surface. Participants achieved different degrees of restricted mobility by wearing soft-soled shoes (S), an ankle-foot orthosis with unrestricted dorsiflexion-plantarflexion activity only (A), and an ankle-foot orthosis with unrestricted dorsiflexion-plantarflexion and adjustable horizontal rotation of the foot (OU/OR). Furthermore, the spatiotemporal parameters, mediolateral margin of stability, center of pressure, angle of the fore and hind foot relative to the tibia, and correlation coefficients of the factors were analyzed. Regression analysis was also performed.

**Results:**

At right heel strike, group A had a significantly lower mediolateral margin of stability than group S and group OU. Meanwhile, forefoot adduction (0.2 < |*r*| <0.4) and plantarflexion (0.2 < |*r*| <0.4), as well as hindfoot internal rotation (0.2 < |*r*| <0.6) and inversion (0.2 < |*r*| <0.4), correlated negatively with lateral stability. Regression analysis revealed forefoot dorsiflexion and supination were the main independent variables for group A. At right heel off, groups OU and OR had a significantly lower mediolateral margin of stability than those in groups A and S. Forefoot adduction (0.2 < |*r*| <0.4) and dorsiflexion (0.4 < |*r*| <0.6) were correlated with lateral stability, as were hindfoot dorsiflexion (0.2 < |*r*| <0.4) and inversion (0.2 < |*r*| <0.4). Regression analysis revealed forefoot abduction and plantarflexion were the main independent variables for groups OU and OR.

**Conclusions:**

The present study verified from gait data that forefoot dorsiflexion and supination at the initial contact of the stance phase were relevant factors for the differences in lateral gait stability, whereas abduction and plantar flexion of the forefoot at the terminal stance phase were the main influencing factors of lateral gait stability.

## 1. Introduction

The frequently occurring traffic accidents, cardiovascular and cerebrovascular events, and the increasing aging of the population in our society have led to the presence of large numbers of potentially or apparently unstable gait holders. Moreover, in the available studies, cases of decreased gait stability or abnormal gait due to disease [1–3] and surgery [4, 5] have been reported. Falls and their secondary injuries caused by instability of gait often have serious consequences. Meanwhile, such consequences also result in significant financial, time, and labor costs associated with care and rehabilitation [6, 7]. Clinical diagnostic and treatment criteria for normal and abnormal gait characteristics allow for timely detection and intervention of gait health conditions in patients with unstable gait, thereby reducing the serious consequences of unstable gait [7].

Gait stability is affected by many factors [8], such as age, walking speed, weight shift, and center of pressure (COP) trajectory. Walking in the living environment is often performed while experiencing complex road conditions, multidirectional disturbances, multitask walking, sound and light stimulation, and other situations that are more complex than those in the laboratory environment [9]. Due to the structure of the human lower limb musculoskeletal system, gait adjustment ability in the sagittal direction is greater than lateral adjustment ability [10]. However, at the same time, lateral adjustment is also considered to be a critical influence on lateral stability.

The scale scores of traditional evaluation methods are subjective, and the static evaluation results cannot fully reflect dynamic stability [11, 12]. Therefore, by using motion capture and other technologies, objective and detailed data are obtained, and gait stability analysis that can distinguish gait events and vector directions can be performed. This is helpful for a simple, unified, and quantitative assessment of the gait stability of people [12]. Biomechanical measurements are relevant for both quantitative assessments of fall risk and gait characteristics in different age populations [13]. Most of the time, in a gait cycle, the projection of the center of mass (CoM) onto the ground is outside the base of support (BoS), but the stability of walking can still be satisfied [14]. The margin of stability (MoS) as one of the gait stability assessment metrics has the advantages of efficiency and simplicity of operation over the local dynamic stability, foot placement estimator, global dynamic stability, and other metrics or methods [15]. Therefore, it is more convenient to be widely used for gait analysis of straight walking and turning. However, due to the variability in the application of MoS, the development of a standard process for the use of the method and the availability of a larger amount of data are needed [16].

Moreover, due to the basic kinematic theories such as inverse dynamics [17] and closed kinetic chain, we can determine the importance of foot and ankle joint action for gait stability. Ankle kinematic parameters have different characteristics in different periods of the stance phase [18]. Therefore, biomechanical gait analysis is of great significance for disease assessment and more targeted treatment plan development. The widespread use of ankle-foot orthoses (AFOs) has provided mobility and stability gains not only for patients with conditions such as cerebral palsy and stroke. In a review of prior studies, there is also a tendency for AFO categories [19] to cause limited joint motion or for AFO stiffness [20] to cause abnormal joint motion in different phases of the walking cycle.

Therefore, in the present study, we observed the changes in biomechanical characteristics and stability of different gait cycles in the stance phase using the limitations and effects that different AFOs possess on the normal joint range of motion and joint movement trends in walking, respectively. The objective was to fill the gap in the observation of the effect of limited foot and ankle mobility on lateral gait stability in prior studies, as well as to provide data on kinematic parameters with MoS as the main factor.

## 2. Method

### 2.1. Participants

Thirty (16 male and 14 female) healthy volunteers participated in the experiment. They were all from Suzuka University of Medical Sciences with a mean age of 20.6 ± 0.8 years and mean height and weight of 1.65 ± 0.02 m and 58.2 ± 2.04 kg. All participants met the following criteria: (1) no psychiatric or neurological disorders or orthopedic disorders that interfere with walking, (2) no cerebellar lesions or bilateral motor deficits, and (3) no dance or gymnastic training for more than three months at any time in their lives.

### 2.2. Ethical Approval

All participants were fully informed and understood the content of this study. All participants confirmed their willingness to participate in the experiment. This study was approved by the Ethics Committee of Suzuka University of Medical Sciences (approval number: 437). This study was conducted following the Helsinki Declaration.

### 2.3. Instruments

The equipment in the laboratory used to obtain kinematic data in the trial included a Motion Capture System (Vicon: Nexus 2.11 and 14 at 100 Hz; Vero v2.2∗12, Vantage 5∗2; Vicon Motion Systems Ltd., Oxford, UK); and five force measurement platforms were used to record three components of ground reaction forces: vector, COP, and the timing of the gait events of heel strike and toe off the ground (AMTI: OR 6-6-OP -2000 force platform; Advanced Mechanical Technology, Inc., Watertown, MA, USA). The following shoes (Figure 1(a)) and ankle-foot orthosis were worn on the participant's right foot: Agilium-freestep orthosis (Ottobock KGaA, Duderstadt, Germany) (Figure 1(b)) and Matsumoto custom orthosis for the right foot (Matsumoto Gishi Co. Ltd., Hayashi Komaki, Japan) (Figure 2(a)). The Agilium-freestep orthosis allows only dorsiflexion and plantarflexion of the foot. The Matsumoto custom orthosis also allows for free dorsiflexion and plantarflexion. And there is a locking hole next to the bottom horizontal rotation axis, which can be adjusted by a locking screw to determine whether to restrict the horizontal rotation (Figure 2(b)).

### 2.4. Experimental Protocol and Data Collection

Participants received instructions before the day of the experiment and practiced at a specific cadence on a 10-m-long linear walking path. Based on the average cadence value of healthy adults in Japan [21], the pace tempo of this experiment was set at 112 steps/min. Participants' weight, height, leg length, knee width, and ankle width were measured and recorded on the day of the experiment. The Oxford Foot Model (OFM), which can provide multisegmental kinematic and kinetic data with accuracy for the study [22], was used based on the need for data on the restricted mobility of the foot and ankle. Therefore, the reflex markers were applied to the skin at the location marked by the OFM method. To prevent high inter-subject variability, an experienced laboratory technician determined the final location of the markers.

Each participant was asked to wear shoes or orthosis on their right foot as follows: S, data while wearing soft-soled shoes; A, gait measurement and recording completed while wearing Agilium-freestep orthosis; S, data collected while wearing soft-soled shoes; OU: gait data with the Matsumoto orthosis but no horizontal rotational restriction holes locked; OR: gait data with the Matsumoto orthosis but the bottom horizontal rotation restriction hole locked. A soft-soled shoe of the same thickness was worn on the left foot. Each participant wore the shoes or AFOs in turn and completed the measurement of gait data for each group of 5 tracks. After one foot and ankle condition was fixed, static modeling was first performed, followed by dynamic data measurements and recording. After data recording for one condition was completed, static modeling and dynamic data measurement and recording for the next foot and ankle condition were performed after an interval of ten minutes.

The Vicon Nexus motion capture data was exported to three-dimensional geometric calculation software (Visual 3D: C-motion), which applied a second-order Butterworth filter with a cut-off frequency of 6 Hz and defined a local coordinate system for each body part. Also, information on spatiotemporal parameters and their normalized means and standard deviations was obtained through Vicon Nexus. FFTBA is the angle between the forefoot segment and the tibial segment, while HFTBA is the angle between the hindfoot segment and the tibial segment. All angles were recorded in the sagittal, frontal, and coronal planes. At least three markers are used to locate each segment. Each gait event was defined and modified to obtain the 3D position coordinate information of the BoS in each gait event and to calculate the MoS. Sincethe CoM trajectory is extrapolated along its velocity direction, theextrapolated center of mass (XcoM) is used for the calculation of MoS. The differencebetween XcoM and the boundary ofBoS is MoS. In this study, the definition of BoS by Ohtsu et al. [23] was followed, and the front boundary and inner boundary of the BoS were defined. The formula for MoS is shown below as Equation (1) and Equation (2). The *x* in the formula is the coordinate of CoM, and *l* is the distance from CoM to the axis of rotation. And *v* is the velocity of CoM. The MoS obtained by this calculation was used as the stability of gait is described by the change in the MoS value. We analyzed the ML MoS of the average of five walking routes for each group for each gait event.

(1) $$\begin{array}{c} \text{MoS}=\text{BoS}-\text{XcoM}, \end{array}$$

(2) $$\begin{array}{c} \text{XcoM}=x+\frac{v}{\omega }=x+\frac{v}{\sqrt{g/l}}. \end{array}$$

### 2.5. Statistical Analysis

The Shapiro-Wilk test was used to examine the distribution and variance of the ML MoS in each group for each walking event, followed by a one-way ANOVA. A post hoc Bonferroni test was then performed to test for significant differences in spatiotemporal parameters, foot and ankle kinematics, ML MoS, and COP based on different ankle-foot mobility limitations. The gait events used for statistical analysis were defined as follows: The time points of right heel strike (RHS), left toe off (LTO), left heel strike (LHS), and right toe off (RTO) were automatically labeled by Vicon Nexus based on data from the force measurement platform. The RTOE at the midpoint of the base of the 1st and 5th metatarsal in the anterior part of the right foot was used to construct the forefoot segment for the calculation of the FFTBA. The vertical coordinates of the RTOE were also used to define the gait event RFF as well as the RHO gait event based on the RFF. The time point at which the velocity of the RTOE is below 100 mm/s was defined as right foot flat (RFF). The right heel off (RHO) was defined when the vertical coordinate of the heel mark is 10 mm or greater than that of the RFF. The moment of immediately coming to LHS was defined as pre-LHS. Significance levels were determined at a 5% risk rate (*p* < 0.05). Statistical analyses were performed using IBM SPSS Statistics 21 statistical software (IBM, Armonk, NY, USA).

## 3. Results

### 3.1. Spatiotemporal Parameters

The results of the spatiotemporal parameter analysis based on one gait cycle are shown in Table 1. The results of the one-way ANOVA and post hoc multiple comparisons showed no significant differences between the results of walking speed and stride length for the following variables. The results of the left foot cadence showed that the values of group A were significantly higher than those of the groups S, OU, and OR (*p* < 0.01). The results of the right foot cadence showed that the values of group A were significantly lower than those of groups S, OU, and OR (*p* < 0.01). In addition, the stride width of group A was also significantly wider than that of groups S and OR (*p* < 0.01).

### 3.2. ML MoS (Mediolateral Margin of Stability)

The results of the analysis of ML MoS in this study showed a significant difference in ML MoS outcomes during the RHS and RHO gait events (Figure 3). The ML MoS values of group A at RHS were significantly smaller than those of groups S and OU (p < 0.05). The ML MoS values in groups OU and OR were significantly smaller than those in groups A and S (*p* < 0.01) at RHO.

### 3.3. COP (Center of Pressure)

According to the normal distribution test results of the Shapiro-Wilk method (*p* < 0.05), the COP results of groups A, S, OU, and OR are all non-normally distributed, so the Kruskal-Wallis (K-W) test was selected. The significant differences in COP were as follows (Figure 4): the values of group A at RHS were significantly greater than those of groups S (*p* < 0.01) and OR (*p* < 0.05); the values of group A at pre-LHS and LHS were significantly smaller than those of group OU (*p* < 0.01) and OR (*p* < 0.05); and the values of group A at RTO were significantly smaller than those of group S (*p* <0.05).

### 3.4. Forefoot Tibia Angle (FFTBA) and Hindfoot Tibia Angle (HFTBA)

The foot tibial angle in a gait cycle is shown below (Figure 5). According to the results of FFTBA and HFTBA, the forefoot adduction angle in group S was greater than in the other three groups during the whole gait cycle, and the forefoot abduction angle in group A was significantly greater than in the other three groups at the end of the stance phase (60%). The forefoot plantarflexion angle of the groups OU and OR in the mid-stance phase was smaller than that of group S, while group A had a greater dorsiflexion angle than the other groups during the whole phase. Moreover, group A showed an opposite dorsiflexion tendency to the other groups at the end of the stance phase. The group OU with unlimited horizontal rotation had greater pronation in the initial contact period, while the range of pronation and supination of the group OR with restricted horizontal rotation was the smallest. The external rotation angle of the hindfoot in group A was smallest in the initial contact phase (0–10%), while its internal rotation angle was smallest in the pre-swing phase (30–60%) than in the other groups. Group S had the greatest hindfoot plantarflexion, while groups OU and OR had the greatest hindfoot dorsiflexion during the whole gait cycle. Group A had the smallest range of inversion and eversion in the standing phase, followed by group OR, which also had no limitation in dorsiflexion and plantarflexion only.

The peaks of the angles of the FFTBA and HFTBA based on the Oxford foot model are shown in Table 2. The groups A, OU, and OR with AFOs exhibited common characteristics of greater forefoot abduction with less adduction, less forefoot plantarflexion, less forefoot pronation, and greater hindfoot dorsiflexion with less plantarflexion than group S. This included the largest forefoot abduction and smallest forefoot plantarflexion in group A, the largest hindfoot dorsiflexion in groups OU and OR, and the smallest hindfoot plantarflexion in group OU. In addition, some disparate features included greater forefoot dorsiflexion and smaller hindfoot internal rotation in group A, smaller hindfoot eversion in groups OU and OR, and greater forefoot pronation in group OU than in group A and OR.

### 3.5. Correlation Analysis and Stepwise Regression Analysis

Since the significant difference in ML MoS appeared at the time of both RHS and RHO gait events, the correlation analysis and stepwise multiple regression analysis of FFTBA and HFTBA relative to ML MoS at these two time points were performed. The values of FFTBA, HFTBA, and ML MOS at RHS and RHO were obtained by Visual 3D. The results of the Pearson correlation coefficient analysis are shown in Table 3.

Stepwise multiple regression analysis of FFTBA and HFTBA concerning ML MoS was implemented.  Figure 6 presents the results of the analysis at RHS, and Figure 7 shows the results of the analysis at RHO.

Each motion angle of the FFTBA and HFTBA at RHS was used as the independent variable (D-W values between 0-4), while ML MoS was used as the dependent variable for stepwise multiple regression analysis. And after automatic model identification, the best-fit equations obtained from stepwise multiple regression analysis can be found in Figure 6.

After automatic model identification, each motion angle of the FFTBA and HFTBA at RHO was used as the independent variable (D-W values between 0-4), while ML MoS was used as the dependent variable for stepwise multiple regression analysis. The best-fit equations obtained from stepwise multiple regression analysis can be found in Figure 7.

## 4. Discussion

The present study showed that different ankle mobility limitations led to differences in lateral stability in different periods of the stance phase. The results showed that participants with limited ankle mobility differed in the spatiotemporal parameters, mainly in terms of changes in cadence and step width. The differences in lateral stability were found at the RHS and RHO. And the COP differences appeared at the RHS, pre-LHS, LHS, and RTO of the stance phase. During the initial contact of the stance phase, the angles of restricted ankle movements mainly associated with poorer lateral stability were forefoot dorsiflexion and pronation, whereas, at the end of the stance phase, the angles of restricted ankle movement mainly associated with poorer lateral stability were forefoot abduction and plantarflexion.

Based on the spatiotemporal parameters, a significant influence of the kinematic parameters received by the foot and ankle in immobilized healthy adults can be found. Parameters such as walking speed and stride length did not differ significantly for participants. However, significant differences were found in parameters such as step width and the cadence of left and right foot. The participant's cadence was significantly lower in the right foot with limited mobility, while the cadence of the contralateral foot was significantly higher. According to prior studies, the step width was also significantly altered, and according to prior studies, this may have occurred as compensation for the limited mobility of the ankle joint [25].

The increase in ML MoS is also considered related to the increase in cadence [26]. As an assessment tool for lateral stability in this study, ML MoS showed significant differences at the RHS and RHO during the stance phase of walking. The difference in ML MoS at the RHS was mainly attributed to the difference in ML BoS. And the difference in ML MoS at RHO was mainly due to the difference in the velocity of lateral movement of the CoM. Therefore, dynamic stability analysis by direction is necessary to improve the sensitivity of fall risk assessment [15, 22].

In comparison with the results of ML MoS, the gait events and groups that showed significant differences in COP were different. The trajectory of COP x in group A showed a greater difference compared to the other three groups. Limited ankle mobility at initial contact can lead to differences in COP and can have an impact on COP during the subsequent stance phase. Mark A et al. [27] assessed the outcomes of treatment for gait deficits using the COP indicator, and the possibility that the change occurred may be based on the improvement of neurofeedback by rehabilitation. In patients with limited ankle mobility, attention can be focused on COP during gait events such as RHS, pre-LHS, LHS, and RTO at the initial and terminal phases of the stance phase.

Based on the contents of Figure 5 and Table 2, the characteristics of FFTBA and HFTBA of each group can be found. The groups (A, OU, OR) with AFOs had the characteristics of small forefoot adduction and large forefoot abduction, which should be attributed to the neutral position design of the AFO. Another characteristic that was widespread across the groups wearing AFOs was a smaller forefoot plantarflexion. This characteristic might well be caused by the AFO's axis of sagittal plane movement deviating from the ankle joint's own axis of dorsiflexion and plantarflexion. Group A's greater dorsiflexion was caused by the AFO's forefoot's lower rigidity. In contrast, the OR group, which allowed only dorsiflexion-plantarflexion and had higher forefoot rigidity, had a significantly smaller range of forefoot pronation and pronation than the other groups. Combined with the results of ML MoS, it is evident that the effect of AFO in preventing sports injuries and proper joint angulation may also create a reduction in lateral gait stability due to joint stiffness [28]. These changes occurred significantly in the initial contact phase and the pre-swing phase when the joint angle changed rapidly.

Correlation coefficient analysis can provide a reference for simplifying the number of observed indicators for stability assessment in the clinical setting. For normal human gait, forefoot dorsiflexion and plantarflexion, and forefoot supination and pronation, as well as hindfoot internal and external rotation at RHS, can be used as the main kinematic parameters to assess the lateral stability of gait. In individuals with no forefoot stiffness but limited pronation-supination and adduction-abduction, forefoot dorsiflexion and plantarflexion at RHS, as well as forefoot abduction-adduction and hindfoot inversion-eversion at RHO, are the main kinematic parameters associated with lateral stability. In individuals with foot stiffness and limited inversion-eversion, pronation-supination at RHS and hindfoot internal and external rotation, as well as dorsiflexion and plantarflexion at RHO, are the kinematic parameters associated with lateral stability. In individuals with foot stiffness with limited adduction-abduction and inversion-eversion, forefoot adduction-abduction, forefoot dorsiflexion-plantarflexion, hindfoot internal and external rotation, and hindfoot inversion-eversion at RHS, as well as forefoot dorsiflexion-plantarflexion and hindfoot inversion-eversion at RHO, are kinematic parameters associated with lateral stability.

The stepwise multiple regression analysis of joint mobility to ML MoS at RHS and RHO provided clues to finding kinetic-related gait stability. At RHS, forefoot supination and forefoot dorsiflexion had a significant positive effect on ML MoS, while hindfoot internal rotation and inversion had a significant negative effect. While at RHO, forefoot adduction and dorsiflexion had a significant negative effect on ML MoS. Based on the *R*^2^ values of the stepwise multiple regression analysis, it can be observed that the variability of the effect of joint mobility on ML MoS was higher in the groups S and A with lower rigidity. In contrast, the variability of the effects of joint mobility on ML MoS was lower in the groups OU and OR, and the optimal regression equation could reflect the true situation with greater probability. Likewise, the stepwise multiple regression analysis of variance was smaller in the single-limb supported phase than in the double-limb supported phase, and the effect of joint mobility on ML MoS was greater.

The inadequate foot pronation and plantar flexion result in inadequate supination of the supporting foot, making the MTP joint tension lower and reducing the rigidity of the Agilium orthosis forefoot support. During this phase, the contralateral limb swings forward over the support foot, generating external rotational forces. This external rotation generates lateral shear forces in the foot that promote rotation back [29]. However, passive supination is accompanied by limited foot mobility; the position of the foot bones that constitute the rigid lever; and the muscles that provide tension for the rigid lever are synergistically poor, resulting in the windlass effect not being fully exploited. Consequently, the stability of the levers, such as the first MTP joint push-off of the foot, is reduced and cannot provide sufficient support height and anterior lateral thrust for the anterior lateral swing of the contralateral swing foot. This disruption of the kinetic chain may be responsible for the lack of antagonistic effects on the control of the CoM transfer velocity. In turn, it affects lateral stability. The deficit in plantar flexion at the end of the stance phase in patients with limited plantar flexion function or the elderly may lead to weak plantar rigidity. This leads to kinetic and kinematic abnormalities, which can affect lateral stability.

For patients with inadequate forefoot control, exercises corresponding to forefoot adduction and abduction, eversion, and plantar flexion [30] should be recommended, or the use of an orthosis that can provide sufficient support for the forefoot to improve the rigidity of the forefoot. Where possible, the functional training of lower limb abductors or extensors and plantar flexors should be strengthened in the neutral position of the hip joint and the hip joint extension position to be closer to the supporting foot function at the vital moments of the stance phase [31]. Therefore, at the end of the stance and before the contralateral heel strike, the forefoot of the supporting foot can be fully internally rotated and vagus, so that the stability of the midfoot joint and the first ray is improved [32], thus providing sufficient support for foot height and joint torque. Consequently, the swinging foot can be fully swung into place to obtain a sufficient BoS; at the same time, so that the CoM shift velocity can be better controlled. In this way, lateral gait stability can be improved [33].

Lateral stability requires active adjustment. And longitudinal stability passive adjustment through the conversion of energy absorbed by the stride and loading response to gradually eliminate external disturbances reduces the impact [4]. In contrast to previous research, this study carried out a correlation analysis of the dynamic indicators in the stance phase as well as an analysis of the differences between the groups according to gait events. In the study of other active factors, the research subjects will adopt an adapted pace, changing their stride length, cadence, etc. based on their exercise ability under specific physiological and pathological conditions, walking tasks, and psychological factors (e.g., fear of falling). Because lateral stability has more active regulation than longitudinal stability, and the frontal control of the foot has a more sensitive influence on lateral stability [34], lateral stability control is of greater significance in dealing with sudden lateral disturbances and preventing the resulting falls [35].

As a widely used rehabilitation treatment for patients, AFO has the effect of improving postural control of the foot and ankle in the swing and loading response phases, which has a significant positive effect on improving gait [36]. However, the restriction of the foot and ankle caused by the AFO can also obstruct the normal degree of movement of the foot and ankle joints. It has been suggested that AFO may impede the advancement of the tibia over the foot during the stance phase and prevent normal gait from occurring [37]. Combined with the results of this study, we suggest that better plantar rigidity combined with a foot adduction-abduction angle appropriate for the wearer may provide better lateral gait stability for the orthotic wearer.

During the transition, gait stability changes, such as loading response and terminal stance phase. This study reveals that the foot responds to loading acceptance primarily with supination and pronation. There is a link between the increase in tendon strain and the ability of the subtalar joint to absorb, and the total pronation [38]. Foot supination can assist in pushing off the ground steadily at the end of the stance phase [30]. In clinical patients with low gait stability or a high incidence of falls, attention should be paid to the patient's ability to perform adduction and abduction of the foot and whether their plantar flexion and supination ability can provide sufficient forefoot rigidity and structural stability of the first ray.

A limitation exists in this study. The model of foot and ankle mobility limitation used in this study was based on normal individuals wearing ankle-foot orthoses. The results of gait characteristics may differ from the effects of joint mobility limitations caused by disease or deformity. Studies based on patients or physically impaired individuals may further validate the reliability of this study.

## 5. Conclusion

This study reveals that lateral gait stability showed significant differences at RHS in initial contact and at RHO in terminal stance under different conditions of limited foot and ankle mobility. The analysis of the groups with significantly low stability during these two gait events indicates that low lateral stability at RHS was positively correlated with forefoot and hindfoot dorsiflexion in the group with transverse and coronal plane restriction as well as low forefoot rigidity. The main positive influence factors of lateral stability were its forefoot dorsiflexion and supination. Low lateral stability at RHO was negatively correlated with forefoot and hindfoot dorsiflexion as well as hindfoot inversion in the group with coronal plane restriction and foot stiffness. The main positive influence factors of lateral stability were forefoot abduction and plantarflexion.

## Figures and Tables

**Figure 1:** Soft‒soled shoes (a) and Agilium‒freestep orthosis (b). The soft-soled shoes have no restrictions on the foot and ankle joints, and the bottom surface is soft and has the same thickness as the orthosis. The bottom surface of the Agilium-freestep orthosis forefoot is soft.

**Figure 2:** Matsumoto custom orthosis (a) and bottom view of the Matsumoto orthosis (b). The bottom surface is hard, which limits the rotation of the forefoot and midfoot to a certain extent. The screw marked by the red circle is the horizontal rotation limiter.

**Figure 3:** The mediolateral margin of stability (ML MoS) during the stance phase. The ML MoS of each gait event during the stance phase. The results in the figure are the mean values of the ML MoS of each group at different gait events (∗*p* < 0.05), (∗∗*p* < 0.01). A:gray column with stripes; S: black column; OU: red column; OR: red column with lattice.

**Figure 4:** Center of pressure (COP) x at each gait event. The figure shows the mean values with SD of the COP x of each group in the different gait events (^∗^*p* < 0.05, ^∗∗^*p* < 0.01). A: gray interrupted lines with dots; S: solid black line with squares; OU: solid red line with triangles; OR: red dotted line with inverted triangles.

**Figure 5:** FFTBA and HFTBA during the gait cycle. (a)–(c) are the results of adduction (ADD) (+)/abduction (ABD) (-), dorsiflexion (DF) (+)/plantarflexion (PF) (-), supination (SP) (+)/pronation (PR) (-) of the FFTBA. (d)–(f) are the results of internal rotation (IR) (+)/external rotation (ER) (-), dorsiflexion (DF) (+)/plantarflexion (PF) (-), inversion (IV) (+)/eversion (EV) (-) [24] of HFTBA. A: black interrupted line, S: black realized, OU: red solid line, OR: red dotted line.

**Figure 6:** Scatter plots of the FFTBA and HFTBA with significant effects on ML MoS and corresponding ML MoS values at RHS. The solid black line is the reference line of the best-fit equation obtained from the stepwise multiple regression analysis.

**Figure 7:** Scatter plots of the joint motion angles with significant effects on ML MoS and corresponding ML MoS values at RHO. The solid black line is the reference line of the best-fit equation obtained from the stepwise multiple regression analysis.

**Table 1:** The result of spatiotemporal parameters (*n* =30).

Variables	A	S	OU	OR
Walking speed (m/s)	1.39 (0.13)	1.41 (0.13)	1.40 (0.13)	1.41 (0.14)
Cadence (steps/min)				
Left	118.75 (4.37)	116.40^∗∗^ (3.50)	116.48^∗∗^ (3.91)	116.20^∗∗^ (4.67)
Right	113.53 (3.92)	116.08^∗∗^ (4.24)	116.79^∗∗^ (4.85)	116.71^∗∗^ (4.27)
Stride length (m)	1.47 (0.12)	1.46 (0.13)	1.46 (0.14)	1.46 (0.14)
Stride width (m)	0.18 (0.02)	0.16 (0.02)^∗∗^	0.17 (0.03)	0.16 (0.02)^∗∗^

Note:^∗^ indicates that the value is significantly different from the value in group A (^∗∗^*p* < 0.01); mean (standard deviation).

**Table 2:** Foot kinematic parameters based on the Oxford foot model (unit: °).

	A	S	OU	OR
*FFTBA*				
ADD	11.2 (6.61) ^##^	18.07 (8.17)	12.65 (6.79) ^##^	11.97 (6.51) ^##^
ABD	-18.05 (7.49)^##^	-6.72 (8.47) ^∗∗^	-13.33 (7.43) ^∗∗^^,##^	-12.2 (6.97) ^∗∗^^,##^
DF	12.67 (5.41)	9.19 (8.25) ^∗∗^	9.69 (5.5) ^∗∗^	8.81 (5.89) ^∗∗^
PF	4.39 (4.3)	0.13 (5.58) ^∗∗^	2.29 (4.42) ^∗∗^^,##^	2.29 (4.99) ^∗∗^^,##^
SP	16.46 (8.28)	16.03 (7.24)	16.38 (7.26)	14.45 (6.8)
PR	8.88 (6.35)	3.61 (5.39) ^∗∗^	5.56 (8.44) ^∗∗^	8.72 (7.72) ^##,$$^
*HFTBA*				
IR	21.98 (8.37)	29.34 (11.87) ^∗∗^	30.28 (6.07) ^∗∗^	29.34 (5.54) ^∗∗^
ER	5.02 (8.94)	4.46 (8.35)	3.28 (7.76)	4.94 (7.34)
DF	4.65 (8.35)	-4.88 (7.29) ^∗∗^	8.8 (8.78) ^∗∗^^,##^	8.72 (7.97) ^∗∗^^,##^
PF	-2.44 (7.97)	-7.48 (7.66) ^∗∗^	0.29 (7.73) ^∗^^,##^	-0.12 (7.14) ^##^
IV	6.72 (10.84)	5.13 (9.0)	9.22 (8.67) ^#^	7.44 (7.81)
EV	1.28 (14.01)	-3.16 (7.97) ^∗^	1.2 (8.68) ^#^	3.09 (16.53) ^##^

Note: ^∗^^,#,$^ indicate significant differences from group A, group S, and group OU, respectively. ^∗^^,#,$^: *p* < 0.05, ^∗∗^^,##,$$^: *p* < 0.01.

**Table 3:** Analysis of the correlation coefficient between FFTBA and HFTBA relative to ML MoS at RHS and RHO.

		FFTBA			HFTBA		
		ADD/ABD	DF/PF	SP/PR	IR/ER	DF/PF	IV/EV
RHS	S	-0.14	0.22^∗∗^	-0.23^∗∗^	-0.35^∗∗^	0.11	-0.31^∗∗^
	A	-0.13	0.30^∗∗^	0.15	-0.09	0.19^∗^	0.05
	OU	-0.16	0.06	0.30^∗∗^	-0.35^∗∗^	0.01	-0.06
	OR	-0.28^∗∗^	0.24^∗∗^	0.14	-0.41^∗∗^	-0.11	-0.31^∗∗^
RHO	S	-0.09	-0.14	0.07	-0.02	0.04	0.07
	A	-0.23^∗∗^	0.01	-0.13	0.13	-0.04	-0.22^∗∗^
	OU	-0.02	-0.56^∗∗^	-0.02	-0.16	-0.22^∗^	0.14
	OR	0.12	-0.65^∗∗^	-0.10	0.16	-0.06	-0.23^∗^

Note: ^∗^ Indicates that the value is significantly correlated with the ML MoS at a given gait event, ^∗^*p* < 0.05, ^∗∗^*p* < 0.01.

## Data Availability

All data used during the study are available from the corresponding author by request “hatanaka@suzuka-u.ac.jp”.
